# The Effect of Introducing Infographic Pattern on Developing Cognitive Understanding by Using AI Technology for University Students during the COVID-19 Pandemic

This article has been retracted.

**DOI:** 10.1155/2021/7197224

**Published:** 2021-10-25

**Authors:** Emad M. Samra

**Affiliations:** College of Computer and Information Systems, Umm Al-Qura University, Mecca, Saudi Arabia

## Abstract

During the COVID-19 pandemic, this study sought to determine the impact of AI-supported infographic templates (static versus animated) on academic achievement, visual thinking skills, and willingness to learn among a sample of university students. The researcher created two distinct AI-supported instructional infographic templates to determine the effect of such an independent variable on his three other primary dependent variables, namely, academic accomplishment, visual thinking skills, and willingness to learn, in order to meet his study goals. An achievement exam, a visual thinking test, and a willingness to learn scale were among the research methods used. The quasiexperimental method was used to provide the research instruments, and experimental therapy was used to a select group of students at Umm Al-Qura University. According to the findings, AI-assisted static and animated infographic templates had a favorable impact on the development of all learning aspects studied. AI-assisted animated infographics, on the other hand, had a more significant impact than AI-assisted static infographics. In light of this, the researcher concluded his research by making a number of recommendations and suggesting additional research, such as maximizing the use of AI emerging technologies and their practical application in an adaptive manner suitable for education.

## 1. Introduction

Emerging digital technology-based environments have significantly contributed to enriching the learning process beyond classroom walls as such drastic change has largely been reflected in all used instructional materials for educational purposes with different features and formats, thus allowing information transfer to learners in various methods and techniques.

In particular, infographic technology is, indeed, one of the most prominent information presentation tools as it empowers users to display required information in an organized way as well as its delivery using different visual stimuli [1]. As previously emphasized in [2], it is necessary to depict and present information at learning environments using visuals as well as take into account differences between various visuals delivering the same information in addition to learners' preferences for obtaining and receiving information.

According to [3], the infographic is a commonly used visual technology for displaying information in a believable manner, allowing for easier comparison of provided data and more clear information presentations. In other terms, an infographic is a visual depiction of complicated concepts and facts that are used to enhance their transmission to a target audience in an efficient and understandable manner. Notably, the infographic is known by a variety of terms, including, but not limited to, visual representation, data visual representation, information design, and information engineering [4–6].

Overall, infographics help students to master 21^st^ century skills as they can be used to serve numerous educational purposes as effective tools for graphic visual representations as well as fast and clear presentation of information, data, or knowledge [7].

Currently, there is ample empirical evidence in the literature repeatedly emphasizing the effective use of infographics in developing students' various cognitive and affective and psychomotor dimensions of learning, e.g., carrying out academic course projects [8], making learning more permanent [9], and facilitating personal learning processes in virtual environments through the construction of audiovisual contents based on graphic design principles [10].

Visual thinking, in a similar vein, is extremely crucial for the learning process. It is used to assist them in resolving problems and assist them in their group work. Such visual thinking tools assist learners in organizing their thoughts and provide a visual aid for depicting the relationship between ideas, facts, or concepts [11].

No wonder then that there is a consensus in the literature on the top priority of supporting the development of visual thinking skills at all K-12 and higher education programs, curricula, and courses, especially among tertiary education students. Notably, several previous studies, e.g., [11–13], concluded a noticeable lack of visual thinking skills mastery among selected samples of students belonging to different educational stages that can be attributed to multiple causes, e.g., inadequate instructional strategies largely based on using traditional old-fashioned teacher-centered teaching methods, instructional materials, curricula, and educational technologies.

In line with these findings, previous research has highlighted the link between effective use of infographics and the development of students' visual thinking skills by encouraging them to be at the center of the learning process and providing them with appropriate training on how to fully utilize their various visual abilities in information retention, analysis, and communication [14–16].

However, to the best of the researcher's knowledge, there have been no previous studies in the literature examining the impact of using various infographic templates as proposed instructional tools for teaching Programming Languages courses on academic achievement, visual thinking skills, and willingness to learn among university students. As a result, there are both theoretical and practical justifications for doing the current investigation.

It is against such backdrop that it is high time for educational infographic templates to cope with and make the utmost use of the latest up-to-date technological innovations in Artificial Intelligence (AI), robotics, machine learning, and big data to enable educators, instructional designers, and curriculum planners and developers to employ infographics as effective data visualization, visual literacy, and instructional tools for teaching and learning 21^st^ century skills in the digital age taking into account the drastic developments, applications, and impacts of the field of Artificial Intelligence in Education (AIED) on administration, instruction, and learning as emphasized in [17].

Moreover, the authors of [18, 19] added that infographics are an important genre of communication, especially nowadays amidst the outbreak of a global pandemic like coronavirus disease 2019 (COVID-19), currently sweeping across the globe, because they not only provide sufficient information and visual messages for communicating health risks, repercussions, and recovery strategies but also do so in an engaging manner in a time of crisis when the mounting fear motivates learners to seek accurate and credible information swifter and also change their health behaviors accordingly.

The next section highlights the problem statement. Then, it is followed by research questions, research hypotheses, aim, and objectives. Next, the research importance, literature review, and research methodology are covered. Beside this, both the stages and steps of designing an educational infographic and determining the visual thinking skills are explained. The research tools, results, and discussion are presented. Lastly, the paper is ended with the conclusion section.

## 2. Problem Statement

As a general rule, the overwhelming majority of faculty members at different universities all over the world are still persistent in relying on using traditional teaching methods from a passive perspective neglecting students' characteristics, interests, attitudes, and inclinations. As a result, the researcher personally realized the fact that if new emerging digital technologies and tools, including AI-supported infographics, are utilized in learning, it will be possible to overcome the chronic problem of providing students with a huge amount of information. Instead, such information can be presented in an attractive visual form making it easy for students to remember, analyze, and transfer at all academic courses.

Practically speaking, in his capacity as a lecturer at Umm Al-Qura University (UQU), the researcher observed a noticeable lack of visual thinking skills and willingness to learn among his Saudi students. Besides, the researcher informally held a number of meetings with some of his college students providing them with the same information presented in both traditional and visual AI-supported infographic versions. Overall, the students confirmed that technologically presented information was better, easier to remember and summarize, and more comprehensible.

More specifically, the researcher specified and formulated the problem of his study in a precise brief statement emphasizing that most academic courses as well as teaching methods, approaches, and strategies currently offered to Saudi university students do neither allow them to master visual thinking skills in practice, nor effectively contribute to developing their academic achievement and willingness to learn.

In light of this, the researcher concluded that identifying and comparing the effect of different AI-supported infographic templates (static versus animated) on developing academic achievement, visual thinking skills, and willingness to learn among a selected sample of Saudi university students is a top priority, especially in light of the COVID-19 pandemic.

## 3. Research Questions

This study attempted to answer the following major question: “*What is the effect of difference between AI-supported infographic templates (static vs. animated) on developing academic achievement, visual thinking skills, and willingness to learn among a sample of students during the COVID-19 pandemic?*”

Then, such question was branched into the following three subquestions that the researcher strived hard to answer, namely,

1. What is the effect of AI-supported infographic, regardless of its templates (static versus animated), on developing academic achievement, visual thinking skills, and willingness to learn among participant students?
2. What is the effect of AI-supported static infographic on developing academic achievement, visual thinking skills, and willingness to learn among participant students?
3. What is the effect of AI-supported animated infographic on developing academic achievement, visual thinking skills, and willingness to learn among participant students?

## 4. Research Hypotheses

This study sought to verify the following six hypotheses:

1. There is a significant difference at the 0.05 level between the mean scores of participant students using AI-supported infographic, regardless of its templates (static versus animated), in the achievement test both before and after application in favor of postapplication
2. There is a significant difference at the 0.05 level between the mean scores of participant students using AI-supported infographic, regardless of its templates (static versus animated), in the visual thinking test both before and after application in favor of postapplication
3. There is a significant difference at the 0.05 level between the mean scores of participant students using AI-supported infographic, regardless of its templates (static versus animated), in the willingness to learn scale both before and after application in favor of postapplication
4. There is no significant difference between the mean scores of the first experimental group students using AI-supported static infographic and the second experimental group students using AI-supported animated infographic in the achievement test
5. There is no significant difference between the mean scores of the first experimental group students using AI-supported static infographic and the second experimental group students using AI-supported animated infographic in the visual thinking test
6. There is no significant difference between the mean scores of the first experimental group students using AI-supported static infographic and the second experimental group students using AI-supported animated infographic in the willingness to learn scale

### 4.1. Research Aim and Objectives

This study has an aim of indicating the different level of effectiveness between AI-supported infographic templates (static versus animated) on developing academic achievement, visual thinking skills, and willingness to learn among a sample of students during the COVID-19 pandemic. To reach this aim, the following three objectives must be accomplished:

1. Designing a double-template educational program to use AI-supported infographic (static versus animated) in teaching Programming Languages course to students at the Department of Information Science, College of Computer and Information Systems, Umm Al-Qura University
2. Verifying the effect of using AI-supported infographic templates (static versus animated) on the research-dependent variables, i.e., academic achievement, visual thinking skills, and willingness to learn
3. Identifying which AI-supported infographic template (static versus animated) has a larger significant effect on the research-dependent variables, i.e., academic achievement, visual thinking skills, and willingness to learn

### 4.2. Research Importance

This study might be of interest to various concerned stakeholders due to its following potential theoretical and practical benefits:

1. Providing a helping hand to assist curriculum planners and developers to make the utmost use of Artificial Intelligence (AI) emerging tools and technologies in the educational process
2. Upgrading learner-centered teaching methods from a more integrated perspective focusing on skills mastery, character formation, self-confidence building and maximizing the spirit of creativity, as prominently emphasized by the Saudi Vision 2030 document
3. If integrated with the results of other relevant research studies, this research results may benefit academic faculty members in planning their lessons in a more effective and interesting way for learners
4. Providing an advanced method for presenting instructional content and materials in a suitable way helping students to form positive attitudes towards learning
5. Opening the door for other researchers, experts, and specialists in both fields of curriculum and educational technology to conduct further relevant studies examining the effectiveness of using AI-supported infographics on developing a multitude of students' desired learning outcomes at different educational stages

## 5. Literature Review

First, although *infographic* use as an instructional material is new, its components are not. In fact, several components, e.g., pictures, drawings, diagrams, symbols, and texts, are usually used to prepare infographics so that they can be utilized either separately or in an integrated manner to present information. There are several Web-based applications (e.g., Piktochart, Canva, ThingLink, Visual.ly, and Infogr.am), graphics editor software (e.g., Adobe Photoshop, Adobe Illustrator, CorelDRAW, and Picasa), and diagram tools (e.g., SmartDraw) that can be used in creating infographics [5].

In general, there are a few different definitions of infographics in the literature. Infographics are short for “information graphics.” The infographic, according to [20], is a coherent visual story made up of graphics. Similarly, an infographic is “a form of visual that integrates facts with design to express messages to its audience,” according to [4]. To put it another way, infographics are visual representations of textual facts, information, and expertise that are designed to make the material presented more accessible and understandable (see Figure 1).

According to [21], the good most powerful infographics include the following four major elements: (1) purpose; (2) style; (3) evidence; and (4) format.

The infographic displays difficult and complex information in an easy and clear way by converting a huge amount of data into images and graphics. Moreover, it grants students the opportunity to compare different sizes, areas, and shapes [14]. Thus, the study in [22] saw infographics as effective knowledge visualization and sharing tools, while the authors of [23] emphasized the significant effect of infographics on promoting information recall as well as the ability to process, memorize, and recall information [4, 24].

Furthermore, the study in [21] illustrated that infographics usually have the following five major characteristics: visual attractiveness; symbolizing and summarizing; ability for sharing; enhancement ability; and enhancing learning process.

The study in [5] found that effective visual communication tools, such as infographics, which are extensively utilized to improve students' memory, should include three key elements. To attract attention and engage an audience, make an appeal. Visual communication requires both comprehension and retention to develop a clear understanding.

In a related vein, the author of [25] identified the following seven principles to be considered when designing and producing any educational infographic.

Specifically, the study in [26] identified three basic types of infographics, each of which is classified based on the multimedia components it contains: static (noninteractive) infographics, animated (semi-interactive) infographics, and interactive infographics are the three types of infographics available.

Second, *visual thinking* is mainly based on the visual/verbal divide [27]. According to the Planning, Attention, Simultaneous, and Successive Processing (PASS) theory of intelligence, there are two different types of cognitive processes that play a pivotal role in determining the way information is coded, transformed, retained, and finally stored in the human brain: simultaneous and successive processing. In simultaneous processing, separate units of information are synthesized into a conceptual group or an integrated whole organization (e.g., processing visual data like diagrams, maps, and graphs). On the contrary, successive processing linearly synthesizes separate units of information into a temporally organized sequence or a chain-like progression (e.g., processing textual data like word order in sentences).

Historically, the study in [28] first derived the “visual thinking” concept in his 1969 classic book of the same title where he equated the acts of thinking and perception by describing the act of perceiving as being much more than simple vision, but, rather, a complex process that is actually thinking. Thus, visual perception allows us to have a true understanding of experience.

However, neurobiologists and physicists have only just begun to comprehend the workings of neural systems that allow images and symbols to interact in the human brain during conscious cognition, thus providing actual physical evidence to further explain the concept of “visual thinking” [29].

Overall, the author of [30] noticed that educational researchers mostly agree that there are (at least) two modes of thought: verbal and visual. Verbal thinking has consistently been considered; visual thinking, in contrast, has often been considered. Visual thinking is the intuitive and intellectual process of visual idea generation and problem-solving [31, 32].

In short, the study in [33] saw visual thinking as an active and analytical process of perceiving. It is processing information through images instead of words. Moreover, it can be seen as using one's visual imagination to take experience and experiment and make new models of reality or using the visual in abstract thought (see Figure 2).

Visual Thinking Strategies (VTS) is a structured arts-based constructivist teaching method that uses strategically selected and sequenced visual art images to encourage students to socially construct knowledge through visual, oral, and written literacy and collaborative discussion. It is based on social learning theory [35].

The author of [36] assumed that the ability to use VTS and understand visual art images develops in five main consecutive stages: accountive; constructive; classifying; interpretive recreative.

VTS ask teachers to facilitate learning through questioning, discussions, learner-centered interactions, observation, and meaning-making. As a result, discussions are facilitated, not directed, by the teacher who motivates student investigation asking three progressively more complex questions to help move students through the stages as shown in [37].

## 6. Research Methodology

This study used the descriptive method to prepare the research theoretical framework, conduct literature review, and design research tools and materials as well as result discussion and interpretation. Besides, the study also used the quasiexperimental method to identify the effect of difference between two AI-supported infographic templates (static versus animated) used in teaching some selected topics at Programming Languages course on developing the research-dependent variables, i.e., academic achievement, visual thinking skills, and willingness to learn, among a sample of university students employing the pretest-posttest experimental group design dividing the research sample (*N* = 60) into two equal experimental groups, each including 30 students (see Table 1 for further details).

## 7. Stages and Steps of Designing an Educational Infographic

The researcher prepared his experimental treatment material, that is, the proposed two AI-supported infographic templates (static versus animated) for developing academic achievement, visual thinking skills, and willingness to learn among the selected sample of university students during the COVID-19 pandemic, going through the following five major successive phases with several substeps:

1. Analysis stage, including analysis of current educational needs, general goal of infographic use as well as learners' characteristics, instructional tasks, and learning environment
2. Design stage, including behavioral and procedural determination of desired instructional objectives, organization of instructional content, identification of infographic good visual design principles and conditions, selection of teaching and learning strategies, and design of evaluation methods, tools, and strategies
3. Development stage, including identification of infographic design software (e.g., Adobe Photoshop, Audacity, GoAnimate, iMovie, Word, and Sound Forge), collection, provision, and production of required multimedia and final production of both AI-supported static and animated infographic templates design prototypes
4. Evaluation stage, including preapplication of the research tools for initial and formative evaluation purposes for exploratory assessment of the efficiency, effectiveness, and quality of both AI-supported static and animated infographic templates design and production before their final field experimentation
5. Implementation stage, including actual usage of both AI-supported static and animated infographic templates in practice via field administration to the selected sample and conducting final summative evaluation through postapplication of the research tools, i.e., achievement test, visual thinking test, and willingness to learn scale

Generally, the researcher followed the educationally standardized procedures for designing e-learning courses and programs repeatedly advocated by various ISD multistage instructional design models and frameworks for designing e-learning experiences, courses, and instructional content in previous literature usually consisting of five consecutive phases: analysis, design, development, implementation, and evaluation [23, 24, 38–40].

More specifically, the researcher employed a plethora of validated principles, criteria, models, and frameworks for the infographics design process in the previous literature proposed, for example, in [1, 11], in preparing his experimental treatment material. In particular, he benefited from utilizing the widely used instructional design model for infographics design, the Nine-Step Process Model for Infographics Design as a theoretical framework guiding his research.

## 8. Determining the Visual Thinking Skills

Visual thinking skills including eight core skills progressively arranged from simple to complex in the following order:

1. *Figure General Visual Reading*. It is the ability to recognize and describe the shape as well as determine its nature and dimensions
2. *Visual Discrimination*. It is the ability to distinguish between the shape and other different shapes in terms of color, size, area, or depth
3. *Information Interpretation*. It is the ability to clarify the implications of words, symbols, and shapes
4. *Information Analysis*. It is the ability to focus on the details and subcomponents of the overall idea of the figure
5. *Relationship Perception*. It is the ability to realize the nature of the cause-effect relationships between various phenomena represented in the figure
6. *Meaning Inference*. It is the ability to formulate concepts, laws, or ideas as well as extract new partial forms from the figure
7. *Visual Closure*. It is the ability to conclude the whole from the sum of its parts or discover the whole in case of missing one or more of its parts
8. *Visual Retrieval*. It is the ability to recall and use visual experiences in new situations

## 9. Research Tools

The researcher used three main validated tools to collect the required data for his current study.

### 9.1. Achievement Test

It assesses participating students' academic progress in a Programming Languages course taught via AI-assisted infographic templates (static versus animated) using Bloom's Taxonomy's first three hierarchical levels, namely, remembering, comprehending, and applying. It consists of 36 questions, 20 true/false, and 16 multiple choice. Psychometric testing was used to confirm its reliability and validity. It has a significant Cronbach's alpha reliability coefficient of 0.84.

Notably, using the independent samples *t*-test for calculating mean score differences between the two experimental groups using both AI-supported infographic templates (static versus animated) in the achievement test before application, it was concluded that the calculated *t*-value (0.785) is nonsignificant. In other words, both groups are equivalent in academic achievement before conducting the experiment and that variable has no prior effect on the experimental treatment (see Table 2).

### 9.2. Visual Thinking Test

It measures participant students' mastery levels of four core visual thinking skills, situation general visual reading, visual discrimination, relationship perception, and visual retrieval, when learning Programming Languages course taught by AI-supported infographic templates (static versus animated). It includes 24 multiple choice items divided into 4 subdimensions. Its reliability and validity were psychometrically verified. For example, it enjoys a high significant Cronbach's alpha reliability coefficient of 0.82 (see Table 3).

Notably, using the independent samples *t*-test for calculating mean score differences between the two experimental groups using both AI-supported infographic templates (static versus animated) in the visual thinking test before application, it was concluded that the calculated *t*-value (0.343) is nonsignificant. In other words, both groups are equivalent in visual thinking skills before conducting the experiment and that variable has no prior effect on the experimental treatment (see Table 4).

### 9.3. Willingness to Learn Scale

It measures participant students' levels of being open to or seeking out new academic topics, experiences, skills, and information that improve their abilities and enjoyment when learning a Programming Languages course taught by AI-supported infographic templates (static versus animated). It includes 20 four-point Likert scale items. Its reliability and validity were psychometrically verified. For example, it enjoys a high significant Cronbach's alpha reliability coefficient of 0.79.

Notably, using the independent samples *t*-test for calculating mean score differences between the two experimental groups using both AI-supported infographic templates (static versus animated) in the willingness to learn scale before application, it was concluded that the calculated *t*-value (0.343) is nonsignificant. In other words, both groups are equivalent in willingness to learn before conducting the experiment and that variable has no prior effect on the experimental treatment (see Table 5).

## 10. Results and Discussion

Following data collection and analysis, the researcher concluded a number of significant results that can be displayed in the following two main sections.

### 10.1. Results for the Effect of Using AI-Supported Infographic Templates (Static versus Animated) on Developing Academic Achievement, Visual Thinking Skills, and Willingness to Learn

To begin, the paired samples *t*-test was used to calculate mean score differences between the two experimental groups in the achievement test both before and after application in order to determine the effect of AI-supported infographic on developing academic achievement, regardless of its templates (static versus animated). At the 0.05 level with 59 degrees of freedom, the estimated *t*-value (39.181) was found to be greater than the tabular value. To put it another way, the mean achievement test results of the two experimental groups differ significantly both before and after application (21.54) and after application (61.26) in favor of the higher postapplication mean scores. Thus, the researcher accepted his study's first hypothesis (see Table 6).

Second, the paired samples *t*-test was used to calculate mean score differences between the two experimental groups in the visual thinking test both before and after application to determine the effect of AI-supported infographics on developing visual thinking skills, regardless of their templates (static versus animated). The estimated *t*-value (23.98) was found to be bigger than the tabular value at the 0.05 level with 59 degrees of freedom. In other words, the mean scores of the two experimental groups in the visual thinking test differ significantly both before and after application (11.800) and after application (24.416) in favor of the higher postapplication mean scores. Thus, the researcher accepted his study's second hypothesis (see Table 7).

Third, the paired samples *t*-test was used to calculate mean score differences between the two experimental groups in the willingness to learn scale both before and after application to determine the effect of AI-supported infographics on developing willingness to learn, regardless of their templates (static versus animated). The estimated *t*-value (21.902) was found to be bigger than the tabular value at the 0.05 level with 59 degrees of freedom. In other words, the mean scores of the two experimental groups in the willingness to learn scale differ significantly both before and after application (13.33) and before application (17.97) in favor of the higher postapplication mean scores. Thus, the researcher accepted his study's third hypothesis (see Table 8).

Overall, the above-mentioned results largely correspond to those repeatedly concluded by several previous studies in the literature emphasizing the significant positive effect of infographics on developing students' academic achievement at various academic subjects and disciplines. It also has an impact on the development of various skills [41, 42], visual thinking skills [14–16], and willingness to learn as well as other related affective learning outcomes like beliefs, perceptions, attitudes, values, emotions, motivation, and self-efficacy [15, 25].

### 10.2. Results for the Effect of Difference between AI-Supported Infographic Templates (Static versus Animated) on Developing Academic Achievement, Visual Thinking Skills, and Willingness to Learn

First, the independent samples *t*-test was used to calculate mean score differences between the two experimental groups in the achievement test after application in order to determine the effect of the difference between AI-supported infographic templates (static versus animated) on developing academic achievement. The estimated *t*-value (6.1) was found to be bigger than the tabular value at the 0.05 level with 58 degrees of freedom. To put it another way, in the achievement test after application, there is a significant difference in mean scores between the first experimental group students using AI-supported static infographic (26.4) and the second experimental group students using AI-supported animated infographic (32.4) in favor of the higher second experimental group students' mean scores. As a result, the researcher rejected his study's fourth null hypothesis in favor of its alternative hypothesis, which states that there is a significant difference in mean achievement test scores between the two groups at the 0.05 level in favor of students in the second experimental group (see Table 9).

Second, the independent samples *t*-test was used to calculate mean score differences between the two experimental groups in the visual thinking test after application in order to determine the effect of the difference between AI-supported infographic templates (static versus animated) on developing visual thinking skills. The estimated *t*-value (4.312) was found to be bigger than the tabular value at the 0.05 level with 58 degrees of freedom. To put it another way, in the visual thinking test after application, there is a significant difference in mean scores between the first experimental group students using AI-supported static infographic (24.2) and the second experimental group students using AI-supported animated infographic (28.1) in favor of the higher second experimental group students' mean scores. As a result, the researcher rejected his study's fifth null hypothesis in favor of its alternative hypothesis, which states that there is a significant difference in the mean scores of both groups in the visual thinking test in favor of students in the second experimental group at the 0.05 level (see Table 10).

Third, the independent samples *t*-test was used to calculate mean score differences between the two experimental groups in the willingness to learn scale after application in order to determine the effect of the difference between AI-supported infographic templates (static versus animated) on developing willingness to learn. The estimated *t*-value (3.6) was found to be bigger than the tabular value at the 0.05 level with 58 degrees of freedom. To put it another way, in the willingness to learn scale after application, there is a significant difference between the mean scores of both the first experimental group students using AI-supported static infographic (43.6) and the second experimental group students using AI-supported animated infographic (48.1) in favor of the higher second experimental group students' mean scores. As a result, the researcher rejected his study's sixth null hypothesis in favor of an alternative hypothesis claiming that there is a significant difference in the mean scores of both groups in the willingness to learn scale in favor of students in the second experimental group at the 0.05 level (see Table 11).

Overall, the above-mentioned results largely correspond to those repeatedly concluded by several previous studies in literature emphasizing that animated infographics usually have more significant positive effects on developing students' various cognitive, affective, and psychomotor learning outcomes than static infographics, for example, facilitating learning complex science subjects [43], promoting information perception, users' interaction and design quality [44], and improving reflective students' academic achievement [45].

## 11. Conclusions

In light of his study results, the researcher finally provided the following recommendations and suggested further research.

### 11.1. Research Recommendations

- To make the best use of utilizing Artificial Intelligence (AI) emerging technologies and their practical application in an adaptive manner suitable to education
- To give priority to visual learning due to its tremendous effect on promoting information retention and rapid recall abilities
- To provide faculty members with advanced in-service training and professional development sessions focusing on various AI-supported infographic design templates and their effective use in all university courses

### 11.2. Suggested Further Research

- To examine the effect of using AI technologies on students' various learning outcomes
- To investigate the effect of current research variables on other students belonging to different colleges and disciplines
- To tackle the effect of other infographic templates on current research-dependent variables, that is, academic achievement, visual thinking skills, and willingness to learn
- To conduct similar studies focusing on different instructional content at other educational stages in light of such diverse variables as grade levels as well as students' interests, inclinations, and motivations towards learning different academic topics and disciplines

## Figures and Tables

**Figure 1:** Anatomy of an infographic [4].

**Figure 2:** Meaning of the visual thinking processes model [34].

**Table 1:** Experimental design of the current study.

Group	Preapplication	Experimental treatment	Postapplication
First experimental group (AI-supported static infographic)	Achievement test	Content delivery using AI-supported static infographic	Achievement test
	Visual thinking test		Visual thinking test
	Willingness to learn scale		Willingness to learn scale

Second experimental group (AI-supported animated infographic)	Achievement test	Content delivery using AI-supported animated infographic	Achievement test
	Visual thinking test		Visual thinking test
	Willingness to learn scale		Willingness to learn scale

**Table 2:** Calculated *t*-values for mean score differences between the two experimental groups in the achievement test before application.

Group	*N*	Means	Standard deviation	Standard error	Degree of freedom	Calculated *t*-value	Significance level
First experimental group (AI-supported static infographic)	30	22.14	7.030	1.188	58	0.785	Nonsignificant
Second experimental group (AI-supported animated infographic)	30	20.94	5.682	0.961			

**Table 3:** Relative weights of visual thinking skills.

Number	Skill	Number of questions	Relative weights (%)
1	Situation general visual reading	6	25
2	Visual discrimination	5	20.83
3	Relationship perception	5	20.83
4	Visual retrieval	8	33.33
Overall		24	100

**Table 4:** Calculated *t*-values for mean score differences between the two experimental groups in the visual thinking test before application.

Group	*N*	Means	Standard deviation	Standard error	Degree of freedom	Calculated *t*-value	Significance level
First experimental group (AI-supported static infographic)	30	20.1	5.9	1.06	58	0.343	Nonsignificant
Second experimental group (AI-supported animated infographic)	30	20.63	6.3	1.15			

**Table 5:** Calculated *t*-values for mean score differences between the two experimental groups in the willingness to learn scale before application.

Group	*N*	Means	Standard deviation	Standard error	Degree of freedom	Calculated *t*-value	Significance level
First experimental group (AI-supported static infographic)	30	5.55	2.49	0.45	58	0.343	Nonsignificant
Second experimental group (AI-supported animated infographic)	30	5.31	2.43	0.43			

**Table 6:** Calculated *t*-values for mean score differences between the two experimental groups in the achievement test both before and after application.

Measurement type	*N*	Means	Standard deviation	Standard error	Degree of freedom	Calculated *t*-value	Significance level
Preapplication	60	21.54	6.374	0.762	59	39.181	Significant at the 0.05 level
Postapplication		61.26	6.426	0.768			

**Table 7:** Calculated *t*-values for mean score differences between the two experimental groups in the visual thinking test both before and after application.

Measurement type	*N*	Means	Standard deviation	Standard error	Degree of freedom	Calculated *t*-value	Significance level
Preapplication	60	11.800	1.387	0.179	59	23.98	Significant at the 0.05 level
Postapplication		24.416	4.013	4.014			

**Table 8:** Calculated *t*-values for mean score differences between the two experimental groups in the willingness to learn scale both before and after application.

Measurement type	*N*	Means	Standard deviation	Standard error	Degree of freedom	Calculated *t*-value	Significance level
Preapplication	60	13.33	2.412	0.5	59	21.902	Significant at the 0.05 level
Postapplication		17.97	1.847	0.44			

**Table 9:** Calculated *t*-values for mean score differences between the two experimental groups in the achievement test after application.

Group	*N*	Means	Standard deviation	Degree of freedom	Calculated *t*-value	Significance level
First experimental group (AI-supported static infographic)	30	26.4	4.8	58	6.1	Significant at the 0.05 level
Second experimental group (AI-supported animated infographic)	30	32.4	2.4			

**Table 10:** Calculated *t*-values for mean score differences between the two experimental groups in the visual thinking test after application.

Group	*N*	Means	Standard deviation	Degree of freedom	Calculated *t*-value	Significance level
First experimental group (AI-supported static infographic)	30	24.2	6.698	58	4.312	Significant at the 0.05 level
Second experimental group (AI-supported animated infographic)	30	28.1	8.841			

**Table 11:** Calculated *t*-values for mean score differences between the two experimental groups in the willingness to learn scale after application.

Group	*N*	Means	Standard deviation	Degree of freedom	Calculated *t*-value	Significance level
First experimental group (AI-supported static infographic)	30	43.6	2.4	58	3.6	Significant at the 0.05 level
Second experimental group (AI-supported animated infographic)	30	48.1	4.7			

## Data Availability

The data used to support the findings of this study are available from the author upon request.

## References

[1] Yildirim S., Yildirim G., Çelik E., Aydin M. (2014). Student opinions about infographics design process. *Journal of Research in Education and Teaching*.

[2] Fleming M. L., Levie W. H. (1993). *Instructional Message Design: Principles from the Behavioral and Cognitive Sciences*.

[3] Krum R. (2013). *Cool Infographics: Effective Communication with Data Visualization and Design*.

[4] Smiciklas M. (2012). *The Power of Infographics: Using Pictures to Communicate and Connect with Your Audiences*.

[5] Lankow J., Ritchie J., Crooks R. (2012). *Infographics: The Power of Visual Storytelling*.

[6] Polman J. L., Gebre E. H. (2015). Towards critical appraisal of infographics as scientific inscriptions. *Journal of Research in Science Teaching*.

[7] Meeusah N., Tangkijviwat U. Effect of data set and hue on a content understanding of infographics.

[8] Troutner J. (2010). Infographics defined. *Teacher Librarian*.

[9] Yildirim S. (2016). Infographics for educational purposes: their structure, properties, and reader approaches. *Turkish Online Journal of Educational Technology: Studies and Research*.

[10] Salas Rueda R. A. (2015). Use of infographics in virtual environments for personal learning process on Boolean algebra. *Revista de Comunicación Vivat Academia*.

[11] Jber Y. S. (2010). Effect of using the metacognitive learning cycle strategy on developing concepts and visual thinking skills in science among tenth-grade basic education students.

[12] El-Sayed‬ S. A. (2011). A proposed program in mathematics designed according to brain-based learning theory to develop academic achievement and some thinking skills among preparatory stage students. *Journal of Suez Faculty of Education*.

[13] Tafesh E. A. (2011). Effect of a suggested program in mathematical communication skills on developing academic achievement and visual thinking skills in geometry among eighth-grade basic education female students in gaza.

[14] Darwish A. M., El-Dakhakhny A. A. (2015). Web-based Infographic templates (static vs. animated) and their effectiveness in developing visual thinking skills among autistic children and their attitudes towards autism. *Educational Technology: Studies and Research*.

[15] Omar A. M. I. (2016). Effectiveness of a proposed strategy based on infographics in acquiring scientific concepts, developing visual thinking skills and enjoying learning science among fifth-grade primary students. *Journal of Scientific Education*.

[16] Al-Rashidi H. A. (2021). Effect of using a training program based on infographic technology on developing academic achievement and visual thinking skills among students of College of Education at University of Ha’il. *Journal of Education, Sohag University*.

[17] Chen L., Chen P., Lin Z. (2020). Artificial intelligence in education: a review. *IEEE Access*.

[18] Jacob R. (2020). Visualising global pandemic: a content analysis of infographics on COVID-19. *Journal of Content, Community and Communication*.

[19] Egan M., Acharya A., Sounderajah V. (2021). Evaluating the effect of infographics on public recall, sentiment and willingness to use face masks during the COVID-19 pandemic: a randomised Internet-based questionnaire study. *BMC Public Health*.

[20] Matrix S., Hodson J. (2014). Teaching with infographics: practicing new digital competencies and visual literacies. *Journal of Pedagogic Development*.

[21] Davis M., Quinn D. (2013). Visualizing text: the new literacy of infographics. *Reading Today*.

[22] Antonova A. (2016). Building sophisticated infographics as effective knowledge visualization and knowledge sharing tool. *Rhetoric and Communication e-Journal*.

[23] Waller K., Hill N., Meyers C., McCord A., Gibson C. (2020). The effect of infographics on recall of information about genetically modified foods. *Journal of Agricultural Education*.

[24] Dunlap J. C., Lowenthal P. R. (2016). Getting graphic about infographics: design lessons learned from popular infographics. *Journal of Visual Literacy*.

[25] Çifçi T. (2016). Effects of infographics on students achievement and attitude towards geography lessons. *Journal of Education and Learning*.

[26] Afify M. K. (2018). The effect of the difference between infographic designing types (static vs. animated) on developing visual learning designing skills and recognition of its elements and principles. *International Journal of Emerging Technologies in Learning*.

[27] Bateman J. A. (2014). *Text and Image: A Critical Introduction to the Visual/Verbal Divide*.

[28] Arnheim R. (1969). *Visual Thinking*.

[29] Kindler A. M. (2003). Visual culture, visual brain, and (art) education. *Studies in Art Education*.

[30] Brumberger E. R. (2007). Making the strange familiar. *Journal of Business and Technical Communication*.

[31] Brasseur L. E. (1993). Visual thinking in the English department. *Journal of Aesthetic Education*.

[32] John-Steiner V. (1997). *Notebooks of the Mind: Explorations of Thinking*.

[33] McKim R. H. (1972). *Experiences in Visual Thinking*.

[34] Bilbokaitė R. (2008). Analysis of visual thinking meaning in science education. *Problems of Education in the 21^st^ Century*.

[35] Housen A., Yenawine P. (2000). *Visual Thinking Strategies: Learning to Think and Communicate through Art*.

[36] Housen A. (2001). *Eye of the Beholder: Research, Theory and Practice*.

[37] Yenawine P. (2014). *Visual Thinking Strategies: Using Art to Deepen Learning across School Disciplines*.

[38] Vanichvasin P. (2021). Effects of visual communication on memory enhancement of Thai undergraduate students. *Kasetsart University. Higher Education Studies*.

[39] Al-Mohammadi N. (2017). Effectiveness of using infographics as an approach for teaching programming fundamentals on developing analytical thinking skills for high school students in the city of Makkah in Saudi Arabia. *Global Journal of Educational Studies*.

[40] Hassan A. H. (2021). The effect of infographics on the cognitive skills development (perception and remembering information) of library and information science students in New Valley University: an experimental study. *Scientific Journal of Library, Archives and Information*.

[41] Ibrahem U. M., Alamro A. R., Alamro A. R. (2021). Effects of infographics on developing computer knowledge, skills and achievement motivation among Hail University students. *International Journal of Instruction*.

[42] Bicen H., Beheshti M. (2017). The psychological impact of infographics in education. *Broad Research in Artificial Intelligence and Neuroscience*.

[43] Hassan H. G. (2016). *Designing Infographics to Support Teaching Complex Science Subject: A Comparison between Static and Animated Infographics*.

[44] Locoro A., Cabitza F., Actis-Grosso R., Batini C. (2017). Static and interactive infographics in daily tasks: a value-in-use and quality of interaction user study. *Computers in Human Behavior*.

[45] Ismaeel D., Al Mulhim E. (2021). The influence of interactive and static infographics on the academic achievement of reflective and impulsive students. *Australasian Journal of Educational Technology*.

